# Effect of Endurance Training in COPD Patients Undergoing Pulmonary Rehabilitation: A Meta-Analysis

**DOI:** 10.1155/2022/4671419

**Published:** 2022-09-07

**Authors:** Yingying Li, Weiwei Wu, Xiaoqiao Wang, Lili Chen

**Affiliations:** ^1^Department of Rehabilitation Medicine, Hainan General Hospital (Hainan Affiliated Hospital of Hainan Medical University), Haikou 570311, China; ^2^Rehabilitation Department of Health Center, Hainan General Hospital (Hainan Affiliated Hospital of Hainan Medical University), Haikou 570311, China; ^3^Department of Rehabilitation Medicine, Hainan Cancer Hospital, Haikou 570100, China

## Abstract

**Background:**

The efficacy of endurance training (ET) on patients with chronic obstructive pulmonary disease (COPD) has been controversial. This study was aimed at meta-analyzing the effect of ET in COPD patients undergoing pulmonary rehabilitation.

**Methods:**

The literature retrieval was performed in databases to screen relevant literature. Inclusion criteria were as follows: (1) subjects—COPD patients; (2) inclusion of interventional and control groups; (3) intervention measures—the interventional group received whole-body ET and other lung rehabilitation training, while the control group did not receive intervention or other lung rehabilitation training; (4) outcome indicators which included at least one of the following—6MWD, modified Medical Research Council questionnaire (mMRC), and COPD Assessment Test (CAT); and (5) study type—randomized controlled trials (RCTs). The Cochrane risk-of-bias tool was used to assess the risk of bias. The chi-square test was used to evaluate the magnitude of heterogeneity. Subgroup analysis was used to explore the source of heterogeneity. A funnel plot and Egger's test were used to evaluate publication bias.

**Results:**

The 6MWD in the ET group was significantly higher than that in the control group (MD = 47.20, 95% CI [28.60, 65.79], *P* < 0.00001). Significant heterogeneity (*P* < 0.00001, *I*^2^ = 76%) without publication bias (*P* > 0.05) was noted. Subgroup analysis showed that the 6MWD of the ET group was significantly larger than that of the control group without heterogeneity (*P* = 0.63, *I*^2^ = 0%; *P* = 0.59, *I*^2^ = 0%) in both the no training subgroup (MD = 79.26, 95% CI [72.69, 85.82], *P* < 0.00001) and other rehabilitation training group (MD = 23.64, 95% CI [6.70, 40.57], *P* = 0.006). The mMRC score (MD = −0.72, 95% CI [-1.09, -0.34], *P* = 0.002) and CAT (MD = −6.07, 95% CI [-7.28, -4.87], *P* < 0.00001) of the ET group were significantly lower than those of the control group. There was no heterogeneity (*P* = 0.32, *I*^2^ = 15%; *P* = 0.16, *I*^2^ = 41%).

**Conclusion:**

ET can improve patients' motor function and reduce dyspnea. ET might be incorporated as an important part of lung rehabilitation training.

## 1. Introduction

Chronic obstructive pulmonary disease (COPD) is a common, preventable, and treatable disease characterized by persistent respiratory symptoms and airflow restriction. Exposure to tobacco smoke and air pollutants has been found to be responsible for the abnormalities found in the airway and/or alveolus [1–4]. Epidemiological studies showed that COPD has already become the 3rd most common cause of mortality worldwide [5–7]. It is expected that the global burden of COPD may continue to increase in the coming decades due to the aggravation of air pollution and the aging population [8–10]. Moreover, COPD is associated with decreased exercise endurance that may adversely affect patients' quality of life [11, 12].

Lung rehabilitation is the most effective nondrug treatment for COPD [13] that has been suggested to be a component of the standard treatment for COPD [14, 15]. The comprehensive pulmonary rehabilitation program includes patient assessment, exercise training, education, nutritional intervention, and psychosocial support. In 2007, the lung rehabilitation guidelines of the American Association of Chest Physicians and the American Heart and Lung Rehabilitation Association proposed exercise training as the cornerstone of lung rehabilitation (level of evidence 1A) [16]. Furthermore, endurance training (ET), which is usually carried out in the form of walking, climbing stairs, running, and cycling [17], is an important part of exercise training [18].

The effect of ET on COPD patients has been controversial. Some studies [19] pointed out that ET could alleviate symptoms of dyspnea and enhance patient exercise capacity. However, ET has also been found to be of no benefits for COPD patients [20]. Previous meta-analyses [21] concluded that upper limb ET could not improve lung function but increase 6-minute walking distance (6MWD). However, the study was limited to upper limb ET and failed to clarify the source of heterogeneity. Therefore, heterogeneity occurs due to a lack of strict screening criteria to control the intervention measures. We conducted a meta-analysis to explore the impact of ET in COPD patients undergoing pulmonary rehabilitation.

## 2. Methods

### 2.1. Retrieval Strategy

Literature retrieval was performed using electronic databases, including PubMed, Embase, the Cochrane Library, Web of Science, China Biology Medicine disc (CBMdisc), China National Knowledge Infrastructure (CNKI), and Wanfang from inception to June 2022 without restrictions on language. In addition, the references in the included literature were also reviewed and screened to expand potentially eligible literature. The retrieval strategy adopted a combination of Medical Subject Headings words and free words. Search terms included (chronic obstructive lung disease OR COPD) AND (endurance training or cycling or walking or limb training).

### 2.2. Literature Screening

Inclusion criteria were as follows: (1) subjects—COPD patients; (2) inclusion of interventional and control groups; (3) intervention measures—the interventional group received whole-body ET and other lung rehabilitation training, while the control group did not receive intervention or other lung rehabilitation training; (4) outcome indicators which included at least one of the following: 6MWD, modified Medical Research Council questionnaire (mMRC), and COPD Assessment Test (CAT); and (5) study type—randomized controlled trials (RCTs).

Exclusion criteria were as follows: (1) duplicate publications, (2) non-RCT, (3) inconsistent intervention measures, and (4) key data that were missing and could not be supplemented by contacting the author.

### 2.3. Literature Screening and Data Extraction

The two authors independently screened the literature and extracted and cross-checked the data. In case of any disagreement, an agreement was reached by discussion or consultation with the corresponding author. The data extracted mainly included the following: (1) the basic information included in the study, including the research topic, the first author, the publication time, and the published journal; (2) baseline characteristics, including the sample size of each group, patient age and sex, and others; (3) interventions; and (4) outcome indicators and outcome measurement data. Missing data could be supplemented by contacting the author.

### 2.4. Assessment of Risk of Bias

Two researchers independently evaluated the risk of bias using the Cochrane risk-of-bias tool for RCT. Any disputes were resolved by seeking the opinion of the corresponding author.

### 2.5. Statistical Analysis

RevMan 5.3 software was used for meta-analysis. Mean difference (MD) with 95% confidence interval (CI) was calculated. The interstudy heterogeneity was analyzed by the chi^2^ test (the inspection level was *α* = 0.1), and the combination of *I*^2^ was used to quantitatively analyze the size of heterogeneity. In the presence of *I*^2^ ≤ 50% and *P* ≥ 0.1, mild heterogeneity was considered and the fixed effects model was used for meta-analysis. Otherwise, the random effects model was adopted. Subgroup analysis was used to explore the source of heterogeneity. Publication bias was assessed using the funnel plot and Egger's test. Two-sided *P* < 0.05 denoted statistical significance.

## 3. Results

### 3.1. Characteristics of Included Literature

A total of 2361 articles were retrieved, among which 14 RCTs with a total of 816 patients with COPD were finally included [19, 20, 22–33]. The screening process is shown in Figure 1. The basic information of literature and risk of bias assessment are shown in Table 1.

### 3.2. Comparison of 6MWD between the ET Group and Control Group

A total of 11 articles compared 6MWD between the ET group and the control group. The random effects model (chi^2^ = 42.53, *P* < 0.00001, *I*^2^ = 76%) suggested that 6MWD in the ET group was significantly larger than that in the control group (MD = 47.20, 95% CI [28.60, 65.79], *P* < 0.00001), as shown in Figure 2. The funnel chart (Figure 3) showed no publication bias among the literature (*P* > 0.05).

Subgroup analysis (Figure 4) according to the different intervention methods of the control group was then performed by dividing the publications into the no training subgroup and other rehabilitation training subgroup. In the no training subgroup, the 6MWD in the ET group was significantly larger than that in the control group (MD = 79.26, 95% CI [72.69, 85.82], *P* < 0.00001), and there was no interstudy heterogeneity (chi^2^ = 0.92, *P* = 0.63, *I*^2^ = 0%). In the other rehabilitation training subgroup, 6MWD in the ET group was also significantly larger than that in the control group (MD = 23.64, 95% CI [6.70, 40.57], *P* = 0.006) without interstudy heterogeneity (chi^2^ = 5.60, *P* = 0.59, *I*^2^ = 0%).

### 3.3. Comparison of mMRC Scores between the ET Group and Control Group

Comparisons between the mMRC scores of the ET group and control group were performed by pooling data from 5 documents. No heterogeneity (chi^2^ = 4.73, *P* = 0.32, *I*^2^ = 15%) was noted. The mMRC score of the ET group was significantly lower than that of the control group (MD = −0.72, 95% CI [-1.09, -0.34], *P* = 0.002), as shown in Figure 5. The funnel plot (Figure 6) indicated no publication bias.

### 3.4. Comparison of CAT Scores between the ET Group and Control Group

CAT scores of the ET group and control group were compared in 4 literature. Meta-analysis (Figure 7) using the fixed effects model (chi^2^ = 5.11, *P* = 0.16, *I*^2^ = 41%) showed that the CAT score of the ET group was significantly lower than that of the control group (MD = −6.07, 95% CI [-7.28, -4.87], *P* < 0.00001). No publication bias was found (Figure 8).

## 4. Discussion

Our meta-analysis showed that 6MWD in the ET group was significantly higher than that in the control group, whereas the mMRC score and CAT score were significantly lower than those in the control group. The results indicated that ET could improve motor function and reduce dyspnea in COPD patients. It should be noted, however, that there was interstudy heterogeneity in terms of 6MWD analyzed by the random effects model. In the subgroup analysis, we then eliminated the heterogeneity by using a fixed effects model, which showed consistent result with overall analysis.

Domaszewska et al. [28] suggested that ET might be related to the levels of prooxidants and antioxidants in COPD patients. They compared the maximal oxygen uptake, pulmonary function parameters, blood concentration of biomarkers of oxidative stress, and antioxidant between the ET group and control group. The results indicated that ET could improve the maximal oxygen uptake and lung function in COPD patients. Meanwhile, ET does not induce oxidative stress and oxidant imbalance in COPD patients. McKeough et al. [23] have shown that ET can significantly increase the endurance exercise time and exercise ability of COPD patients. ET combined with strength training can significantly alleviate dyspnea and the rate of perceived exertion in COPD patients. They believed that ET combined with strength training might be suitable for COPD patients receiving community rehabilitation training. Zambom-Ferraresi and colleagues [26] compared the effects of resistance training alone and resistance training combined with ET on COPD patients. The results showed that resistance training alone and ET combined with resistance training had similar effects on 6MWD and quality of life in COPD patients. However, ET was noted to increase patient muscle strength and improve patient endurance performance. They observed reduced heart rate and serum lactate levels but comparable quality of life in patients receiving ET. Furthermore, strength training with upper limb ET has also been demonstrated to significantly improve the quality of life and muscle strength than strength training alone [25]. However, both methods have similar effects in reducing CAT scores. Upper limb ET showed no advantage in reducing dyspnea symptoms. In a study that assessed ET in COPD patients by walking down the slope, improved lung function and quality of life were shown [27]. Compared with the control group, the ET was associated with significantly longer distance on 6MWD and improved motor ability that could antagonize skeletal muscle adverse reactions caused by COPD. Ground walking training could benefit COPD patients, especially in improving lung function and quality of life, as indicated by the fact that patients who received ground walking training had milder symptoms of dyspnea than those who received routine training [24]. However, this finding was disputed in another study that noted no such phenomenon [20]. Although simple walking training could reduce the sedentary time, it had no clinical significance for COPD patients. However, no reasons were explained for the discrepancy between their two studies. Our analysis showed that the difference might be related to the inconsistency of training time and intensity. The work by Breyer et al. [29] showed that Nordic walking for 3 months was feasible in different stages of COPD and could significantly improve patients' standing time, reduce sedentary time, and increase 6MWD, all of which were absent in the control group. The curative effect of Nordic walking still existed 9 months after training. Hernández et al. [22] suggested that the shuttle walk test could improve patients' dyspnea and their quality of life, but it had no significant effect on pulmonary function. Jin et al. [32] found that the CAT score in the ET group decreased from 23.4 to 15.6, and the 6MWD increased from 238.0 m to 386.0 m. The score of mMRC decreased from 3.3 to 2.8, which was significantly better than that of the control group. Quantitative walking exercise training can effectively improve the activity tolerance and quality of life for patients with moderate and severe COPD. Wang et al. [30] showed that 5000-step arm swing exercise could not change the pulmonary function but could significantly improve the quality of life in COPD patients. Li et al. [31] showed that the pulmonary function, 6MWD, and CAT scores were improved after exercise in both groups compared with baseline. However, the improvement was more prominent in the interventional group. Duan et al. [19] showed that patients in the ET group could benefit from the CAT score and 6MWD. In addition, walking training can also reduce the number of acute exacerbations. Zhang et al. [33] have shown that high-intensity exercise training of lower limbs can improve the exercise endurance and ventilation function of patients with stable COPD during exercise, but it has no significant effect on static lung function.

Our research suffers from several limitations. First, the observed high risk of bias in some included publications might confound study results. Second, the intervention methods, training cycle, and frequency in each literature were inconsistent. Different training intensity might have different effects on COPD patients. Third, most literature lacked long-term follow-up data, and we could not clarify the duration of endurance training efficacy. Finally, the changes of 6MWD, mMRC, and CAT scores might also be related to demographics and study design. However, due to the lack of relevant information in the literature, we were unable to elucidate their relationships.

In conclusion, ET can improve patients' motor function and reduce dyspnea. ET might be incorporated as an important part of lung rehabilitation training [19, 20, 22–33].

## Figures and Tables

**Figure 1:** Document screening flow chart.

**Figure 2:** Forest map: comparison of 6MWD between the ET group and control group. 6MWD: 6-minute walking distance; ET: endurance training.

**Figure 3:** Funnel plot that compares 6MWD between the ET group and control group. 6MWD: 6-minute walking distance; ET: endurance training.

**Figure 4:** Subgroup analysis forest map: comparison of 6MWD between the ET group and control group. 6MWD: 6-minute walking distance; ET: endurance training.

**Figure 5:** Forest map: comparison of MMRC between the ET group and control group. mMRC: modified Medical Research Council questionnaire; CAT: COPD Assessment Test; ET: endurance training.

**Figure 6:** Funnel plot that compares MMRC between the ET group and control group. mMRC: modified Medical Research Council questionnaire; CAT: COPD Assessment Test; ET: endurance training.

**Figure 7:** Forest map: comparison of CAT between the ET group and control group. CAT: COPD Assessment Test; ET: endurance training.

**Figure 8:** Funnel plot comparing CAT between the ET group and control group. CAT: COPD Assessment Test; ET: endurance training.

**Table 1:** Literature review and risk bias assessment.

Author	Year	Language	No. of patients		Outcomes	Risk of basis
			ET	Control		
Breyer [29]	2010	English	30	30	6MWD	Low risk
Domaszewska [28]	2022	English	20	12	mMRC	Uncertain
Duan [19]	2016	Chinese	46	40	6MWD; CAT	High risk
Hernández [22]	2000	English	20	17	6MWD; mMRC	Uncertain
Jin [32]	2016	Chinese	48	38	6MWD; mMRC; CAT	High risk
Karagiannis [25]	2021	English	18	18	mMRC; CAT	Uncertain
Li [31]	2015	Chinese	50	50	6MWD; CAT	High risk
McKeough [23]	2012	English	16	14	mMRC	Uncertain
Moezy [27]	2018	English	14	16	6MWD	Low risk
Wang [30]	2015	Chinese	23	23	6MWD	Uncertain
Wootton [20]	2017	English	77	44	6MWD	Uncertain
Wootton [24]	2014	English	62	39	6MWD	Uncertain
Zambom-Ferraresi [26]	2015	English	14	8	6MWD	Low risk
Zhang [33]	2012	Chinese	19	10	6MWD	Uncertain

6MWD: 6-minute walking distance; mMRC: modified Medical Research Council questionnaire; CAT: COPD Assessment Test; ET: endurance training.

## Data Availability

The data used to support the findings of this study are available from the corresponding author upon request.
